# A Low-Cost, Autonomous Gait Detection and Estimation System for Analyzing Gait Impairments in Mice

**DOI:** 10.1155/2021/9937904

**Published:** 2021-11-12

**Authors:** Pranav U. Damale, Edwin K. P. Chong, Sean L. Hammond, Ronald B. Tjalkens

**Affiliations:** ^1^Department of Electrical and Computer Engineering, Colorado State University, Fort Collins, CO 80523-1373, USA; ^2^Division of Clinical Pharmacology and Toxicology, University of Colorado, Anschutz, CO 80045-2608, USA; ^3^Department of Environmental and Radiological Health Sciences, Colorado State University, Fort Collins, CO 80523-1601, USA

## Abstract

With the advancement in imaging technology, many commercial systems have been developed for performing motion analysis in mice. However, available commercial systems are expensive and use proprietary software. In this paper, we describe a low-cost, camera-based design of an autonomous gait acquisition and analysis system for inspecting gait deficits in C57BL/6 mice. Our system includes video acquisition, autonomous gait-event detection, gait-parameter extraction, and result visualization. We provide a simple, user-friendly, step-by-step detailed methodology to apply well-known image processing techniques for detecting mice footfalls and calculating various gait parameters for analyzing gait abnormalities in healthy and neurotraumatic mice. The system was used in a live animal study for assessing recovery in a mouse model of Parkinson's disease. Using the videos acquired in the study, we validate the performance of our system with receiver operating characteristic (ROC) and Hit : Miss : False (H : M : F) detection analyses. Our system correctly detected the mice footfalls with an average H : M : F score of 92.1 : 2.3 : 5.6. The values for the area under an ROC curve for all the ROC plots are above 0.95, which indicates an almost perfect detection model. The ROC and H : M : F analyses show that our system produces accurate gait detection. The results observed from the gait assessment study are in agreement with the known literature. This demonstrates the practical viability of our system as a gait analysis tool.

## 1. Introduction

Gait impairments are one the most common traits of many neurodegenerative diseases, such as Parkinson's disease (PD), multiple sclerosis, amyotrophic lateral sclerosis, Huntington's disease, and spinal cord injury. Many human neurological diseases are studied using their mouse models [1]. Since preclinical mouse models of these diseases replicate their respective gait abnormalities [2], gait analysis in mice has always been a topic of interest for gaining insight into neurodegenerative diseases and identifying potential treatments. While validated commercial systems for gait analysis in mice exist, they remain expensive and use patented or proprietary implementation of unpublished work. To address the need for an economic gait assessment system, in this paper, we describe a design for a low-cost monitoring and assessment system for mice gait that can provide the necessary data comparable with some of the commercial systems already available in the market.

Traditionally, gait analysis in mice has been performed through visual inspection [3] and open field activity monitoring [4]. With advancements in imaging technology, many commercial systems have been developed for monitoring mice gaits, such as Animal Strideway Systems (Tekscan, Inc., South Boston, MA, USA), DigiGait Imaging Systems (Mouse Specifics, Inc., Framingham, MA, USA), and CatWalk XT (Noldus Information Technology, Wageningen, NL). There even have been individual attempts to develop an independent gait analysis system, such as one made by Casey Harr of the University of Kentucky [5]. The Animal Strideway System uses thin-film force sensors for gait acquisition combined with digital imaging software for displaying the results. The DigiGait Imaging System implements a treadmill with a transparent treadmill belt and digital imaging hardware and software. CatWalk XT uses a glass trackway equipped with image capturing hardware and software for gait assessment. All these systems provide possible options for gait acquisition in their own right, but they remain quite expensive and are protected with patents that apply closed source implementation.

In recent years, there has been a growing literature on examining the gait kinematics in rodents during preclinical trials. In [6], Maghsoudi et al. proposed a superpixel-based image segmentation method to examine the kinematics of running rodents to improve our understanding of motion control and to aid in treating motor impairments. The method utilizes spatial and color information for image segmentation to extract various features from the images. Wong and Shah [7] proposed a method to collect and analyze three-dimensional kinematics data of quadrupedal locomotion in rodents for preclinical trials. Their method utilizes a six-camera motion capture system to analyze the gait in rodents during treadmill locomotion and studies a variety of motion behaviors in healthy and neurotraumatic rats. In [8], Timotius et al. suggested a gait analysis technique that systematically scales individual gait parameters in mice and rats based on their video-derived silhouette length and area data along with body weight and age. The silhouette-scaled parameters are used for identifying the body length independent motor functional differences in transgenic Huntington's disease mice and PD rats. An open-source gait analysis suite called GAITOR [9] studies gait pattern changes in rodents during preclinical trials. The GAITOR suite is capable of detecting gait changes in rodent models of monoiodoacetate (MIA) injection of joint pain, sciatic nerve injury, elbow joint contracture, and spinal cord injury.

These efforts provide viable solutions for acquiring gait kinematics data in rodents. The gait kinematics data is useful for examining certain aspects of the gait, such as the position of joints and segments through each phase of the gait. However, these are not the only gait parameters indicative of neurodegenerative disease. Quantitative gait pattern analysis used during preclinical trials calculates parameters such as cadence, stance, step and duty cycle, and interleg coordination. Available commercial systems for assessing these gait pattern parameters remain expensive.

To address the need for a cost-effective, robust system for comparing gait abnormalities in mouse models of neurological diseases to a baseline or control group, we have developed and built an inexpensive, camera-based system for gait acquisition and assessment using an LED-lit glass trackway. We have also independently developed algorithms for the extraction of various gait metrics and their analysis, which are implemented using MATLAB R2015b (MathWorks, Inc., Natick, MA, USA). Our system autonomously detects the gait and extracts a large set of kinematic parameters, such as positioning of footfalls, step patterns, contact and noncontact gait metrics, and interleg coordination. While we restrict our attention to the development and performance of these algorithms in this paper, a detailed build of our system is given in [10].

We validate the accuracy of our gait detection algorithms with a receiver operating characteristic (ROC) analysis performed during a live animal study assessing recovery in a classical murine model of PD. We also calculate the Hit : Miss : False (H : M : F) ratio to verify the accuracy of our gait detection system during the same study. The study was conducted over a period of two weeks in three groups of C57BL/6 mice. The first group was administered with Saline. The second group was dosed with methyl-4-phenyl-1,2,3,6-tetrahydropyridine (MPTP), which induces motor impairments identical to those observed in PD. The third group was treated with MPTP and 1,1-bis(3′indolyl)-1-(p-chlorophenyl)methane (C-DIM12), which has demonstrated efficacy in reducing MPTP-induced neuronal loss in mice [11–14]. The experimental setup and the training and habituation of mice to the trackway are explained in detail in [15]. Various gait metrics data acquired during the study showed general agreement with the known literature.

Apart from studying neurodegenerative diseases with the help of gait analysis, there is a wide variety of real-world problems that can be solved using accurate gait detection and estimation. Gait recognition at a distance is useful for video surveillance [16–19]. Characteristic gait parameters, such as varus instability in the knee or ankle at heel strike, are useful to perform comparisons between disguised perpetrators and suspects. Remote gait detection and analysis can be used for healthcare monitoring [20–22]. Gait is a good indicator of our overall health status. Remote gait analysis can be effectively used to support the healthcare needs of the elderly in a noninvasive and reliable manner. Also, the unique gait features of a person can be used for biometric identification along with traditional methods such as fingerprint, face, or iris recognition [23–26]. Gait biometrics identifies features of an individual walking style, such as the shape and gesture, and is one of the recent biometrics systems. Clearly, systems analyzing gait patterns in daily life are in demand due to their noninvasive nature and ease of application.

Gait recognition is implemented as a combination of multiple techniques, such as object localization, motion recognition, and spatiotemporal event detection. Object localization refers to identifying the location of one or more objects in an image and drawing a bounding box around their extent. Motion recognition is the process of detecting a change in the position of an object relative to its surroundings or a change in the surroundings relative to an object. Events that can change in both time and space are called spatiotemporal events. Spatiotemporal event detection is used to model dynamic events such as animal movement and traffic control. The most popular approach for human gait recognition is the use of video recordings, where different methods, such as silhouette-based gait recognition and gait feature extraction, are implemented for identifying moving objects in the video [27–34]. Another approach is the use of wearable sensors, where gait data is collected by the sensors attached to the person's body or limb [35–42]. Yet another approach is the use of thermal sensors, where infrared thermal imaging is used for collecting human gait data and to remove noises from the complex background [43–45]. All these efforts highlight the growing interest gait recognition has gained from researchers and the need for an inexpensive, easy-to-implement system that can be reliably used for accurate gait detection and estimation.

The main contribution of this paper is to provide a step-by-step process for building a gait acquisition system and describe the necessary image-processing algorithms for autonomous gait detection and parameter extraction. We also provide the gait analysis results using our described system from a live animal study that validates the efficacy of the system. A lack of open-source information is one of the major limiting factors for building a low-cost gait analysis system. Gait analysis is one of the nonintrusive ways of diagnosis. The healthcare industry is experiencing a state of revolution with modern computers providing faster diagnosis and therapeutics. Despite modern electronic equipment and computers getting cheaper each year, healthcare remains expensive in all parts of the world. The detailed build guide provided in [10] and the image-processing algorithms provided in this paper mitigate this limiting factor, enabling implementation of an inexpensive gait analysis system.

The remainder of this paper is organized as follows. In Section 2, we give a detailed description of the gait acquisition and detection algorithms used in our system. In Section 3, we present detection performance, ROC analysis, and gait assessment results of the system performed during an in-lab experimental study. We discuss the overall performance and potential improvements of our system in Section 4 and provide concluding remarks in Section 5.

## 2. Method

Our gait acquisition system consists of a long trackway across which a single mouse can run and algorithms to detect the position and pressure of footfalls. The trackway is two meters long and is made of glass, with a rectangular enclosure, a ventrally located camera to capture footfalls, top- and side-mounted LEDs, and a computer with our data processing algorithms and a graphical user interface (GUI) developed in MATLAB. The rectangular enclosure is made of plastic and is placed on the top of the glass trackway to ensure that the mouse continues to run in a particular direction during an experiment. The goal of the system is to autonomously detect and analyze the gait characteristics of the mouse for the experiment.  Figure 1 shows the proposed gait acquisition system, and Figure 2 shows an overview of the gait acquisition and assessment process. Each component is further discussed in detail in the following sections.

### 2.1. Video Acquisition

LEDs are mounted on the top and side of the glass trackway to illuminate the footfalls of the mouse. Red LEDs are installed on the inside of the top side of the rectangular enclosure, and green LEDs are installed along the sides of the glass trackway. The LEDs are equipped with adjustable intensity dimmers. The red LEDs illuminate the glass trackway in a red glow. The light from the green LEDs is reflected internally everywhere inside the glass trackway, except at those areas where the footfalls of the mouse make contact with the glass. The green light is refracted towards the camera at the footfalls creating a strong contrast between the footfalls and the background. This is illustrated in Figure 3. A high-end camera provides a high sampling rate and resolution, both of which are extremely important in collecting gait data. A higher-resolution camera helps in capturing relatively fine details of the footfalls of a mouse, while a higher frame rate ensures that no footfalls are missed while recording a video. The camera of choice was GoPro HERO3+ (GoPro, Inc., San Mateo, CA, USA), which can be installed easily on the adjustable mount to determine the exact field of view of the lens. The videos are recorded at 60 frames per second (fps) and 1080 × 1920-pixel resolution with the help of the GoPro remote user interface. The captured videos are transferred to a computer and are processed using MATLAB with the help of the Image Processing and Computer Vision Toolbox.

Once the videos are acquired, we need to perform some preprocessing on the image sequence before we acquire the gait data. The primary aim of data preprocessing is to extract only the necessary parts of an image and to avoid any extra processing for faster analysis. Also, we need to adjust for any possible distortion or rotation present in an image. For these purposes, we use the system GUI for manually setting the parameters for the preprocessing. First, we load an image from a video to be analyzed. Second, we use the system GUI to remove any barrel distortion in the image. Third, we rotate the image to make sure that the trackway is oriented horizontally in the image. Last, we mark the top and bottom walls of the glass trackway to crop the image to a fixed dimension and to remove the unnecessary areas. Figures 4 and 5 demonstrate the preprocessing steps applied to a sample image. The preprocessing parameters are saved using the system GUI and will be applied to the rest of the image sequences automatically as part of the preprocessing routine.

### 2.2. Paw Detection

In general, any digital image consists of a rectangular grid of pixels, where a pixel is the smallest controllable element of an image represented on the screen. In the RGB color imaging system, color is generally represented by the three-component intensities, namely, Red, Green, and Blue. A major task in paw detection is differentiating the pixels in an image representing the footfalls of a mouse from the rest of the pixels in that image. This task is simplified when there is good color contrast between the pixels representing the footfalls and the rest of the pixels. The previously described LED lighting for the gait acquisition helps in creating such contrast. Differentiating these pixels is achieved by detecting the pixels with sufficiently high green (*G*) values in an RGB image. More specifically, it is adequate to detect the pixels with sufficiently high *G* values within the rectangular enclosure in an image of the glass trackway. At the beginning of the analysis, the top and bottom ends of the rectangular enclosure are manually set from a random frame in the video. To avoid detecting any possible noise, we use the thresholding technique to ensure that only the pixels representing the mouse's footfalls are differentiated.  Algorithm 1 summarizes this technique.

After thresholding for the *G* value, there are still many pixels remaining in the image which need to be identified as paws or otherwise. Proximity clustering, which links closely related pixels to form a larger object, is used for joining the digits of the paws together which are disjointed from the palm area. The distance between two pixels located at 2D positions *p* and *q* is measured by the Euclidean norm, represented by ‖*q* − *p*‖. Pixels within a predefined threshold distance are then grouped. This is summarized in Algorithm 2.

Finally, the clusters that are assumed to be paws, but are smaller or larger than some predefined thresholds, are filtered out. This eliminates the clusters formed by unwanted areas such as noise, dust, and mouse feces on the glass trackway. This procedure is summarized in Algorithm 3.

After finalizing the paw clusters, the centroids of these clusters are recorded for each frame of an acquired video. The set of *N* pixels belonging to cluster *k* at the frame *t* is denoted as *p*_*k*_*t*__={*p*_*k*_1,*t*__, *p*_*k*_2,*t*__,…, *p*_*k*_*N*,*t*__}, with coordinates of pixel *p*_*k*_*i*,*t*__ at *t* being (*x*_*i*_, *y*_*i*_). Here, the *X* direction is along the trackway, while the *Y* direction is perpendicular to the trackway. The centroid for cluster *k* at time *t* is

(1) $$\begin{array}{c} C_{k_{t}}=\frac{1}{N}\sum_{i=1}^{N}p_{k_{i,t}}. \end{array}$$

The centroid represents a 2D location of the paw cluster at a given time.

Figure 6 depicts two sample images from a test video after the application of Algorithms 1–3. Our system correctly identifies two paw clusters in Figure 6(a) and four paw clusters in Figure 6(b). The system automatically marks the detected paw clusters with bounding boxes and also indicates their positions inside the image by highlighting their respective *X* and *Y* coordinates. Later, in Section 3.1, we show that our system very rarely misses a paw cluster present in an image or falsely identifies some area in an image as a paw cluster. In Section 3.2, we explain how to choose particular threshold values in Algorithms 1–3 and how they affect the false alarms and missed detections. The system saves these values of *X* and *Y* coordinates for all detected paw clusters along with their respective frame numbers for further classification.

### 2.3. Paw Classification

The detected paw clusters need to be classified into four groups, namely, *Left-Front*, *Right-Front*, *Left-Rear*, and *Right-Rear*. There is a minimum of one and a maximum of four paw clusters present in each frame, and these paw clusters need to be matched with their corresponding paws in the previous and future frames. There may also be a mouse's tail or nose detected in some frames in addition to some random noise that may be present. This redundant data needs to be eliminated. The main difficulty with the paw classification is that the rear paws often occupy similar locations that the front paws have previously occupied. This leads to many repeated coordinate entries in the recorded data even for different paws.

To solve this problem, first, we categorize the images from a video by the number of paw clusters detected in each frame. In the frames with four paw clusters, classification of individual clusters into *Left-Front*, *Right-Front*, *Left-Rear*, and *Right-Rear* is fairly easy. These are usually the frames where a mouse is standing on all four of its paws. The classification is done by using the *X* and *Y* coordinates for the detected paw clusters. Given the fixed left to the right direction with which a mouse is allowed to run on the trackway, the two clusters with higher *X* coordinates are classified as the front paws, and the remaining two are classified as the rear paws. The front and the rear paws are then further classified into the left and right paws based on their *Y* coordinates. The fixed direction of the mouse movement ensures that the right paws are the ones with the smaller *Y* coordinates and vice versa. This is summarized in Algorithm 4.

We move recursively from the frames with classified paw clusters to their previous and successive frames. Any unclassified paw cluster within a predefined threshold distance from a classified paw is assigned to the same category as that of the classified paw. This is summarized in Algorithm 5. The process is repeated until there are no more new classifications. The remaining unclassified clusters at the end of this process are eliminated as redundant data. The thresholds for the distance and the frames were determined based on a large number of trial runs and cross verification.

### 2.4. Parameter Extraction

Various gait parameters can be calculated from the classified paws. These gait parameters are useful for tracking any irregularities in gait. The gait parameter definitions commonly used in clinical gait analysis are listed for the reader's convenience in Table 1. These definitions are used by the CatWalk XT system and are only used to guide our system's proper estimation of these parameters.

#### 2.4.1. Run Duration

The GoPro HERO3+™ camera is able to capture frames at a rate of 60 fps. The run duration (RD) is calculated as

(2) $$\begin{array}{c} RD=\frac{\left|t_{f}-t_{l}\right|}{60}, \end{array}$$

where *t*_*f*_ and *t*_*l*_ are the times of the first and last frames with at least one detected paw.

#### 2.4.2. Step Recognition

To compute the gait parameters, the steps must first be recognized accurately. The *X* coordinates of each classified paw are projected into a *Distance versus Time* graph as shown in Figure 7. Each run is composed of two phases: *Contact phase* as recognized by the horizontal line parts and *Swing phase* as recognized by diagonal line parts. The number of steps *S* is obtained directly from the number of contact phases during one entire run. The cadence (Cad) is calculated as

(3) $$\begin{array}{c} \mathrm{Cad}=\frac{S}{\text{RD}}. \end{array}$$

#### 2.4.3. Stride Length, Swing Duration, Stance, and Duty Cycle

Let *t*_*f*_^*j*^, *t*_*m*_^*j*^, and *t*_*l*_^*j*^ represent first, mean, and last frames, respectively, for step *j*, and let the centroids associated with step *j* for a particular paw be *C*_*t*_*f*_^*j*^_, *C*_*t*_*m*_^*j*^_, and *C*_*t*_*l*_^*j*^_. Now stride length is calculated as

(4) $$\begin{array}{c} L_{j}=\left\|C_{t_{m}^{j}}\left(x,y\right)-C_{t_{m}^{j+1}}\left(x,y\right)\right\|, \end{array}$$

and the *average stride length* for a particular paw is calculated as

(5) $$\begin{array}{c} L=\frac{1}{S}\sum_{i=1}^{S}L_{i}. \end{array}$$

The *swing duration* is calculated as

(6) $$\begin{array}{c} D_{j}=\frac{\left|t_{l}^{j}-t_{f}^{j+1}\right|}{60}, \end{array}$$

and the *average swing duration* for a particular paw is calculated as

(7) $$\begin{array}{c} D=\frac{1}{S}\sum_{i=1}^{S}D_{i}. \end{array}$$

The *stance* is calculated as

(8) $$\begin{array}{c} R_{j}=\frac{\left|t_{f}^{j}-t_{l}^{j}\right|}{60}, \end{array}$$

and the *average stance* for a particular paw is calculated as

(9) $$\begin{array}{c} R=\frac{1}{S}\sum_{i=1}^{S}R_{i}. \end{array}$$

Once swing duration and stance are obtained, the *duty cycle* is calculated as

(10) $$\begin{array}{c} \mathrm{DC}=\frac{\sum_{i=1}^{S}R_{i}}{\sum_{i=1}^{S}R_{i}+\sum_{i=1}^{S}D_{i}}. \end{array}$$

#### 2.4.4. Paw Support

Paw support indicates the relative duration of simultaneous contact of two or more limbs with the trackway. Different paw supports as defined in Table 1 are calculated by comparing the frame numbers for the steps of the required paws. Once we get the shared frames for the paws, we obtain the duration of their simultaneous contact simply by adding the total number of shared frames and dividing it by 60.

#### 2.4.5. Paw Pressure

Paw pressure is represented in the form of an image by creating a surface plot for the green pixel values in a paw cluster. Smoothing of the curve is achieved by interpolating the values using a spline filter. The area of a paw cluster is calculated as the total number of green pixels in a paw cluster. The *average area* for a particular paw is then calculated as the mean of areas of all the paw clusters of the same category. The intensity of a paw cluster is calculated as the mean of green pixel values in a paw cluster. The *average intensity* of a particular paw is then calculated as the mean of intensities of all the paw clusters of the same category.

### 2.5. Visualization

The system GUI provides all control options and shows visualization results on the extracted gait parameters. Visualizations for some of the gait parameters acquired during the live animal study are shown in Figures 8 and 9. Visualization plays an important role in the quick and efficient analysis of large data. The system GUI can also be used to save the analyzed data in *.mat* or *.csv* formats for future use.

## 3. Results

The system described above was used during a live animal study as one of the tools for assessing the recovery in C57BL/6 mice acquired from Charles River Laboratories (Wilmington, MA, USA), which were medically induced with PD using MPTP and treated with C-DIM12. The study started with three different groups, each consisting of 12 healthy mice, and was conducted over a period of 14 days. The first group was treated with *Saline* throughout the experiment. The second group was injected with *MPTP* on days 1, 5, 9, and 13. The third group was treated with MPTP on the same days, along with oral gavage of C-DIM12 compound dissolved in corn oil (or corn oil vehicle control). On the 14th day, the mice were terminated. Behavior was assessed at these time points using the gait acquisition system. The detailed training and habituation of mice to the trackway is given in [15]. After the treatment, each mouse was allowed to run on the trackway with optimally present lightning. The trackway was wiped with alcohol solution after each run to clean any excretion left by the mice during a run. Each mouse was allowed to run twice for the sake of obtaining better test results. A run with the least number of stops was selected for the analysis using the gait detection system. A total of 328 videos or approximately 196,800 frames were analyzed using our system.

From the video analysis, we acquired the footfall dataset for each frame in the video in terms of the categories *Left-Front*, *Right-Front*, *Left-Rear*, and *Right-Rear*, as well as *X* and *Y* coordinates for each footfall indicating the centroid of the footfall. Algorithms 1–3 detect footfalls in the video and return a set of *X* and *Y* coordinates associated with the footfalls along with their respective frame numbers. Algorithms 4 and 5 classify the detected footfalls into the appropriate categories *Left-Front*, *Right-Front*, *Left-Rear*, and *Right-Rear*. To label the footfalls, we used a graphical image annotation tool called LabelImg [46]. LabelImg is an open-source tool written in Python and uses Qt for its graphical interface. First, we annotated every footfall in each frame of the video with its correct paw class and *X* and *Y* coordinates. Then we saved the annotations in XML files using LabelImg. After saving the annotations, we cross-referenced the gait detection data acquired using our autonomous gait detection algorithms with the annotated gait data using LabelImg as described above. Finally, we used the system GUI to extract the gait parameters as defined in Table 1.

In this section, we show the results for the evaluation of the gait detection algorithms using H : M : F detection ratio, ROC analysis, and gait metrics acquired for the gait assessment.

### 3.1. Hit : Miss : False Detection Ratio

H : M : F detection ratio is the ratio of the percentage of positive paw identification (hit) to missed paw identification (miss) to false identification (false). A *positive* paw identification denotes correct identification and classification of paws present in each frame. A *missed* detection is when the system fails to detect one or more paws present in any frame. A *false* detection is incorrect identification of an object as a paw or misclassification of a detected paw. The goal of the gait acquisition and detection system is to generate close to 100% positive detection.

A missed detection can be caused by low contrast between a paw and the glass trackway. This happens when the area where a paw makes contact with the glass plate is not illuminated enough to be detected through the paw detection threshold explained in Algorithm 1. It may also happen when a paw is being lifted, and the area of the contact is so small that it does not get detected through the threshold in Algorithm 3. A missed detection causes a gap in the acquired gait data and can compromise the recorded gait metrics.

A false detection can be caused by some random noise or a large enough object other than a paw to be falsely labeled as a paw cluster. Most commonly it is caused by a mouse's nose or tail making contact with the glass trackway. False detection can also mean misclassification of some detected paw clusters. This usually happens when a mouse is trying to turn on the trackway during a run, making Algorithm 4 incorrectly classify one or more of the detected paw clusters.

We allowed the system to perform autonomous gait detection and paw classification as explained by the algorithms given in the previous section. For evaluation, we manually labeled all the footfalls present in each frame. Our described system correctly detected and classified each footfall across all the frames with an average H : M : F score of 92.1 : 2.3 : 5.6. The minimum H : M : F score was 84.3 : 0.9 : 14.9, where a large number of footfalls were misclassified due to the mouse turning in the opposite direction midway through a run. The maximum H : M : F score was 96.0 : 1.4 : 2.6, where the mouse completed a near-perfect run with minimum stops.

### 3.2. Receiver Operating Characteristic Analysis

To evaluate how the system performs with the various threshold values for the variables used in Algorithms 1–3, we did an ROC analysis for each of these algorithms.

The gait detection system performs the role of a binary classifier by analyzing each pixel in each image of a video and returning a value of positive or negative for whether the pixel is a part of a paw cluster or not. For the ROC analysis, we chose a test set of carefully selected images from multiple videos. These images represent different possible scenarios while a mouse is walking on the glass trackway: all paws were present, only two paws were present, and so forth. After performing gait detection on the test set for each threshold, we analyzed the accuracy of gait detection using the manually labeled data. For the system performing as a binary classifier with a given threshold, there are four possible outcomes. Each correctly detected paw cluster is counted as “true positive (TP),” incorrectly detected paw cluster as “false positive (FP),” missed detection of a paw cluster as “false negative (FN),” and the rest of the pixels as “true negative (TN).” In each image, only the center part of the image consisting of the glass trackway was analyzed, making it a total of 1720 × 70 possible positive and negative pixels in an image. Each bounding box of TP, FP, and FN is assumed to have a size of 20 × 20 pixels, and the rest of the pixels are labeled as TN. The *true-positive rate (TPR)* for the classifier with a given threshold is then estimated as

(11) $$\begin{array}{c} \mathrm{TPR}\approx \frac{\mathrm{TP}}{\mathrm{TP+FN}}. \end{array}$$

The *false-positive rate (FPR)* of the classifier is

(12) $$\begin{array}{c} \mathrm{FPR}\approx \frac{\mathrm{FP}}{\mathrm{FP+TN}}. \end{array}$$

ROC curves depict how a model's TPR (shown on the vertical axis) varies as a function of its FPR (shown on the horizontal axis). For a binary classifier, each threshold value corresponds to a single point (i.e., (FPR, TPR) pair) in the ROC plane. Conceptually, we may imagine varying threshold values for a variable from −*∞* to +*∞* and tracing a curve through ROC space. Computationally, this is not an optimal way of generating an ROC curve [47]. Instead, an (empirical) ROC curve for each variable in Algorithms 1–3 is constructed by computing FPR and TPR at each threshold value, varied within a reasonable finite range, and interpolating by drawing a straight line between points corresponding to consecutive thresholds. The area under an ROC curve (AUC) is a commonly used summary statistic, typically ranging between 0.5 (random model) and 1 (perfect model) [48].

The ROC curves for Algorithms 1 and 2 are shown in Figures 10(a) and 10(b), respectively, while Figures 11(a) and 11(b) depict the ROC curves for the minimum and maximum cluster size obtained using Algorithm 3. We can see that the AUC values for all the plots are above 0.95, which indicates an almost perfect detection model. Here, we also show the optimal threshold (OT) values in each ROC plot which achieved the maximum TPR and minimum FPR for the respective ROC curve. Then we construct confusion matrices for each of the OT values. The confusion matrices for the green pixel threshold, proximity cluster threshold, minimum cluster size, and maximum cluster size are shown in Figures 12(a), 12(b), 13(a), and 13(b), respectively. The confusion matrices show that there were 0 FN detections for each of the OT values and the maximum FPR was 0.028 for the maximum-cluster-size threshold. Again, all these confusion matrices indicate that the performance of our described gait detection algorithms was near perfect.

### 3.3. Experimental Gait Analysis

The gait analysis system was used to assess locomotor function in the different mice groups during the experiment. The analysis showed an increase in stance period and run duration for the mice treated with MPTP, which were largely restored to control levels by day 13 in mice treated with MPTP + C-DIM12. The comparison of stance period and run duration between the three groups is shown in Figures 8(a) and 8(b), respectively. Stride length analysis also showed significantly shorter rear limb stride lengths in the MPTP group compared to stride lengths in the MPTP + C-DIM12 group from day 9 onward. The change in stride lengths for Left-Rear and Right-Rear paws is shown in Figures 9(a) and 9(b), respectively. The detailed gait analysis results are presented in [15]. Another recent study utilized the stride length calculated using our described system as one of the indicators to show that chronic exposure to Manganese is associated with neuroinflammation and extrapyramidal motor deficits resembling features of PD [49]. The values obtained for these gait metrics are in good agreement with the known literature [50–53]. These results show that our system can be reliably used to indicate gait abnormalities in mice.

## 4. Discussion

Quantitative gait analysis in mice during preclinical trials has always been one of the go-to methods for studying neurodegenerative diseases, such as PD or Huntington's disease. The commercial systems available in the market for such gait analysis are expensive and implement patented software. To address this issue, we developed an economic rodent gait analysis system. A detailed build guide for constructing this low-cost system is provided in [10]. In this work, we described the necessary image-processing algorithms for accurate gait detection and estimation. Our system autonomously detected and classified mice gait with very high accuracy when compared to the manually labeled actual footfalls. The gait metrics data acquired during the experiments indicate the robustness of the system for assessing mice gait abnormalities. The average processing time for one video using our described algorithms is approximately five minutes; thus, it can replace the time-consuming efforts of manual labeling and measurements. Overall, our system has the potential to offer a cost-effective, autonomous gait assessment tool that can be used for studies involving tracking disease progression related to locomotor function and planning treatment strategies.

### 4.1. Economic Factors

We reiterate that our main goal is to build an economic gait analysis system that can provide a reliable alternative to the commercial systems available in the market. The typical cost of a commercial system for gait analysis in rodents is around $50,000. With the help of the detailed build guide described in [10] and the gait detection and estimation algorithms described in this paper, a robust gait analysis system can be built for under $5,000. This cost includes an academic license for MATLAB. Although our software was written in MATLAB, the purpose of this paper is to describe the underlying gait analysis algorithms. Indeed, our algorithms are also easily implemented in open-source systems such as Python. The system can be upgraded even further as needed by replacing the camera module, though prices for these high-speed, high-resolution cameras vary widely (≈$1,000–$25,000). Nonetheless, our described system provides a viable option for constructing a reliable gait analysis system under 10% of the cost of commercial systems.

### 4.2. Current Limitations

There are a few limitations to our described gait detection algorithms. One limitation is the dependence of Algorithms 1–3 on adequate lighting conditions at the time of recording to create sufficient contrast between the mice footfalls and the rest of the image. Inadequate lighting conditions at the time of recording result in difficulty detecting all footfalls present in the videos, which cause loss of data and incorrect gait parameter calculations. This can be rectified by recording multiple sample videos before the actual experiment to ensure that the lighting conditions are adequate. Another limitation is that Algorithm 4 relies on the mouse moving in the designated left-to-right direction. If the mouse turns in the opposite direction midway through a run, the footfalls might be misclassified, resulting in incorrect gait parameters. To avoid such scenarios, all mice in our experiments were trained and habituated to the trackway [15]. Algorithm 5 relies on a predefined threshold to correctly associate unclassified footfalls with those of correctly classified footfalls. We determined this threshold manually to minimize the number of unclassified paw identification. Still, in certain scenarios, some detected footfalls might not be identified, resulting in loss of data and incorrect gait parameter calculations. We can trade off the probability of correctly identifying footfalls with that of false alarms by updating the threshold value in Algorithm 5. Overall, by training and habituating the mice to the trackway, ensuring the lighting conditions are adequate at the time of video acquisition, and, updating the threshold value in Algorithm 5, we remedy the limitations of our described gait detection algorithms for reliable gait detection and estimation.

### 4.3. Future Scope

To further improve the results, one can easily replace the existing camera with an improved camera that can capture videos at a higher resolution and frame rate. In practice, the supporting threshold values for Algorithms 1–3 need to be adjusted for optimal autonomous gait detection. With better-resolution cameras, the detection algorithms can be improved to approach the ultimate goal of a 100 : 0:0 H : M : F detection score. Also, with faster computing processors and optimized software implementation, one can achieve real-time video processing. The GUI can be modified as desired. Finally, machine learning techniques can be implemented for assessing irregularities in the mice gait. This is part of our ongoing study.

## 5. Conclusions

In this paper, we have described a low-cost gait acquisition and analysis system for assessing gait abnormalities in mice. Our system automatically detects mice footfalls and calculates gait parameters, such as cadence, stride length, and bodyweight distribution. Using this system, we were able to extract various gait parameters to track the progression of PD in groups of mice under controlled dosages of a drug. We validated the detection performance of the system by performing an ROC analysis and calculating H : M : F detection ratio. The ROC and H : M : F analyses show that our system produces accurate gait detection. The results observed from the gait assessment study are in agreement with the known literature. This shows that our system can be reliably used for further studies involving mice gait abnormalities related to disease progression and treatment strategy.

## Figures and Tables

**Figure 1:** Gait acquisition system.

**Figure 2:** System overview.

**Figure 3:** A sample image of the trackway, zoomed-in, to show the illuminated footfalls.

**Figure 4:** Application of the preprocessing steps to a sample image. (a) Original image. (b) Image after correcting for barrel distortion.

**Figure 5:** Application of the preprocessing steps to a sample image. (a) Image after correcting for rotation. (b) Cropped image showing just the glass trackway.

**Figure 6:** Sample images showing detected paws after application of Algorithms 1–3. (a) Image with two detected paw clusters. (b) Image with four detected paw clusters.

**Figure 7:** Distance travelled by each paw during a sample run.

**Figure 8:** Graphical visualization of gait parameters for the live animal study. (a) *Stance period* for the three mice groups on the 13th day. (b) *Run duration* for the three mice groups on the 13th day. Error bars indicate 95% confidence intervals calculated over 20 measurements in 24 videos (*n* = 480).

**Figure 9:** Graphical visualization of gait parameters for the live animal study. (a) Change in *stride length* for the *Left-Rear* paw. (b) Change in *stride length* for the *Right-Rear* paw. Error bars indicate 95% confidence intervals calculated over 20 measurements in 24 videos (*n* = 480).

**Figure 10:** ROC curves with the optimal threshold (OT) values for (a) green pixel threshold and (b) proximity cluster threshold.

**Figure 11:** ROC curves with the optimal threshold (OT) values for (a) minimum cluster size and (b) maximum cluster size.

**Figure 12:** Confusion matrices for (a) green pixel threshold = 205 and (b) proximity cluster threshold = 2.

**Figure 13:** Confusion matrices for (a) minimum cluster size = 65 and (b) maximum cluster size = 510.

**Algorithm 1:** Green pixel threshold.

**Algorithm 2:** Proximity clustering.

**Algorithm 3:** Cluster sizing.

**Algorithm 4:** Four-paw classification.

**Algorithm 5:** Unclassified paw identification.

**Table 1:** Definitions of gait parameters.

Parameter	Definition
Run duration	Time of finishing an entire run
Stride length	Distance between two consecutive travels in the same paw
Swing duration	Duration of no contact of a paw with the glass
Swing speed	Ratio of the stride length to the swing duration
Stance	Time the paws are in contact with the glass
Step cycle	Time between two consecutive initial contacts of the same paw
Duty cycle	Percentage of the stance over the sum of the stance and the swing duration
Cadence	Number of steps per time interval in the trial
Base of support	Distance between the fore limbs and the hind limbs at the maximum area
Diagonal dual support	Relative duration of simultaneous contact of two limbs with the glass
Three-point support	Relative duration of simultaneous contact of three limbs with the glass
Four-point support	Relative duration of simultaneous contact of four limbs with the glass
Average area	Average area of a paw contacting the glass
Average intensity	Average pressure of a paw contacting the glass

## Data Availability

Previously reported gait analysis data were used to support this study and are available at DOI: 10.1124/jpet.117.246389 and DOI: 10.1093/toxsci/kfaa115. These prior studies are cited at relevant places within the text as references [11, 14], respectively. The video recordings for the mice gait data used to support the findings of this study are available from the corresponding author upon request.

## Abbreviations

PD: Parkinson's disease
ROC: Receiver operating characteristics
MPTP: Methyl-4-phenyl-1,2,3,6-tetrahydropyridine
C-DIM12: 1,1-Bis (3′indolyl)-1-(p-chlorophenyl)methane
H : M : F: Hit : Miss : False
GUI: Graphical user interface.
